This article has been retracted.

# Early Diagnosis of Brain Injury in Premature Infants Based on Amplitude-Integrated EEG Scoring System

**DOI:** 10.1155/2021/6684818

**Published:** 2021-03-15

**Authors:** Xinyuan Guo, Yanfang Geng, Lei Zhang, Shiping Niu, Jiang Xue

**Affiliations:** ^1^Department of Neonatology, The Second Hospital, Cheeloo College of Medicine, Shandong University, Jinan, Shandong, 250033, China; ^2^Huantai County Maternal and Child Health Care Hospital of Zibo City, Zibo, Shandong, 256400, China; ^3^Zaozhuang Maternal and Children's Hospital, Zaozhuang, Shandong, 277100, China; ^4^Zibo Maternity and Child Health Care Hospital, Zibo, Shandong, 256400, China

## Abstract

Analyzing and discussing the relationship between brain injury in preterm infants and related risk factors can provide evidence for perinatal prevention and early intervention of brain injury in preterm infants, thereby improving the quality of life of preterm infants. This paper selects term preterm infants diagnosed with preterm infant asphyxia in the NICU of a university's First Affiliated Hospital from January 2018 to February 2019 as the research object. In addition, healthy term infants born at the same time in the obstetric department of this hospital are selected as the control group. Both groups of premature infants were monitored for brain function within 6 hours after birth. The aEEG results range from background activity (continuous normal voltage, discontinuous normal voltage, burst suppression, continuous low voltage, and plateau) and sleep-wake cycle (no sleep-wake cycle, immature, and mature sleep-wake cycle) to epileptic activity (single seizures, recurrent seizures, and status epilepticus), three aspects to judge. Statistical analysis uses SPSS 17.0 software. Amplitude-integrated EEG is a simplified form of continuous EEG recording. The trace of the trace represents the voltage change signal of the entire EEG background activity, which can reflect the EEG amplitude, frequency, burst-inhibition, and other pieces of information. aEEG can reflect the degree of HIE lesions in premature infants and the long-term prognosis. It is easy to operate and effective in diagnosis and can be continuously monitored. It is worthy of clinical popularization. There is a good correlation between the expression of EEG and biomarkers. Combining multiple methods can diagnose HIE earlier and evaluate the prognosis.

## 1. Introduction

With the improvement of modern perinatal medicine and intensive care of preterm infants, the survival rate of preterm infants, especially those with very low and ultralow birth weight, has been increasing year by year, and the mortality rate has been decreasing year by year [1, 2]. However, premature birth is still the leading cause of death in premature infants and the second cause of death in children under 5 years of age. The quality of life of premature infants with a perinatal brain injury has become the focus of attention of the whole society [3]. There are two main types of brain injury in premature infants, namely, intracranial hemorrhage and periventricular white matter softening. Severe brain damage in premature infants can lead to death or moderate-to-severe neurodevelopmental disorders, including cerebral palsy, mental retardation, and vision and hearing impairment, and seriously affect the quality of life of preterm infants [4, 5]. Therefore, the early evaluation and prevention of brain injury and its adverse neurological prognosis in preterm infants have become the focus of medical research in preterm infants.

Imaging examinations are of great significance in the diagnosis and evaluation of brain damage in preterm infants [6]. Although both head color Doppler ultrasound and MRI have predictive value for poor neurological prognosis of preterm infants, there are still some preterm infants with neurodevelopmental disorders and imaging examinations did not find brain injury changes. At present, aEEG has been widely used to monitor the brain function of preterm infants with term asphyxia, and aEEG abnormality can be used as an early predictor of hypoxic-ischemic encephalopathy in term infants [7]. However, the application of aEEG in preterm infants is not universal. Recent studies have shown that abnormalities of aEEG are related to brain damage and poor neurological prognosis in preterm infants [8]. Early postnatal monitoring of aEEG provides a valuable time window for neuroprotective intervention. The aEEG of a normal-term premature infant presents a wide and narrow continuous band. The wideband represents quiet sleep, and the narrowband represents active sleep or wakefulness. Different from normal-term infants, the normal aEEG background activity of very premature infants is discontinuous and undergoes a developmental process from immature to mature [9]. With the increase of maturity, the duration of low-voltage activity is shortened, the duration of the outbreak increases, and the amplitude of the outbreak decreases. Therefore, the background activity gradually becomes continuous in the awakened state. Sleep-wake cycles can be seen in babies who are in good condition at 25-26 weeks of gestational age [10]. Starting from 30 to 31 weeks, the QS period can be clearly distinguished on the aEEG graph, which is manifested as an increase in bandwidth, which lasts 20–30 minutes [11]. The classification system created by related scholars classifies the results of aEEG into 3 categories according to the upper boundary, lower boundary amplitude, and presence or absence of epileptiform activity. This classification method is mainly used to evaluate term premature infants or normal premature infants. Researchers have proposed a classification method of EEG background activity, based on EEG terminology, including the classification of sleep-wake cycles that can be used in all preterm infants [12–14]. These two classification methods are complementary to each other and can evaluate the aEEG of premature infants well. Therefore, this study combined these two methods to analyze the results of aEEG in preterm infants. Imaging examination has become a routine examination in the intensive care unit of preterm infants, and head ultrasound is still the first choice for diagnosing brain injury in preterm infants [15]. However, the assessment and prediction of prognosis of brain injury in premature infants by cranial ultrasound require dynamic monitoring results [16]. Previous studies have reported that the sensitivity and specificity of cranial ultrasound for predicting poor neurological prognosis in preterm infants ranged from 45% to 90% [17]. Related scholars conduct bedside monitoring of preterm infants with encephalopathy to observe their EEG background activities to guide the diagnosis and treatment of convulsions and encephalopathy in premature infants. They believe that the data coupled with MRI examination can improve the detection of seizures and encephalopathy in term infants and can predict short-term prognosis [18–20].

The behavioral function of premature infants is not sound, and the value of clinical examination in evaluating neurodevelopment is limited. EEG is more sensitive than some clinical indicators in reflecting brain function and can be used to evaluate the maturity of brain development and determine the severity of brain injury. In this study, a premature infant with full-term asphyxia was the object of study. aEEG was recorded within 6 hours after birth, combined with clinical symptoms and imaging examination (cranial CT or MRI), to observe the correlation between aEEG and the degree of asphyxia. The diagnostic value of brain injury in early infants with perinatal asphyxia and the significance of assessing recent organ damage provide a theoretical basis for early diagnosis and early intervention for early infants with a brain injury after perinatal asphyxia. Amplitude-integrated EEG is a kind of brain function monitoring equipment for premature infants developed in recent years. It has the advantages of noninvasiveness, bedside operation, intuitive graphics, easy early long-term continuous monitoring, and easy interpretation, which greatly improves real-time monitoring, identification, and prognostic judgment of brain injury in critically premature infants. In this paper, aEEG was tested in premature infants with hypoxic-ischemic encephalopathy, and the value of aEEG in early diagnosis and prognostic evaluation of hypoxic-ischemic encephalopathy in premature infants was further discussed.

The rest of this paper is organized as follows.  Section 2 analyzes the high-risk factors related to brain injury in premature infants.  Section 3 gives information and methods.  Section 4 discusses the experimental results.  Section 5 summarizes the full text.

## 2. Analysis of High-Risk Factors Related to Brain Injury in Premature Infants

### 2.1. PVL Classification and Pathology of Premature Infants

Periventricular leukomalacia (PVL) of premature infants is one of the most characteristic forms of brain injury in premature infants. It is related to secondary cerebral palsy and mental retardation, which seriously affects their later motor development and quality of life. PVL is generally divided into two types, cystic PVL and noncystic PVL. Cystic PVL is the deep focal necrosis of periventricular white matter accompanied by the destruction of all cellular components and may show cystic lesions after a few weeks; noncystic PVL lesions are diffusely distributed in the periventricular white matter. It is related to glial cells, microglia, and oligodendrocytes. The severity of PVL lesions adopts de Vries grading method.

- Grade I: periventricular local echo enhancement (PVE) lasts or exceeds 7 days, and no cystic cavity injury occurs thereafter.
- Level II: local echoes around the ventricles are enhanced, and then they turn into local small cyst cavity injury.
- Grade III: extensive echo enhancement around the ventricle is enhanced and then turns into extensive cystic cavity injury.
- Grade IV: extensive echo enhancement around the ventricle is enhanced, involving the subcortical white matter, and then transformed into diffuse cystic cavity injury around the ventricle and subcortex.

Among them, grade I refers to noncystic PVL, and grade II and above PVL is also called cystic PVL. Cystic PVL is more common in grade II PVL, followed by grade III PVL, and grade IV PVL is rare. Reports on the incidence of PVL at all levels vary from country to country. The overall study shows that the total incidence of PVL including noncystic PVL is about 19.8%–34.1%, and the incidence of cystic PVL is 2.5–23.0%. The schematic diagram of the mechanism of PVL is shown in Figure 1.

PVL mainly occurs in the terminal blood supply part of the long perforating artery, and it is commonly located in the peripheral white matter of the triangle and occipital angle of the lateral ventricle (optical area, the terminal blood supply area of the long perforating branch of the middle cerebral artery and the posterior artery). Pathological findings showed that, 6–12 hours after the occurrence of acute hypoxia-ischemia, under the microscope, coagulative necrosis of the white matter first appeared in the periventricular injury site, the necrotic cells showed uniform periodic acid-Schiff (PAS) staining positive and normal structure, and the axon at the edge of the necrosis was swollen obviously, followed by different degrees of necrosis and loss of oligodendrocytes constituting the axon myelin sheath, so the axon broke and softened foci formed. About 24 to 48 hours later, microglia infiltration appeared at the necrotic site, accompanied by the proliferation of mast astrocytes and endothelial cells. About 5 days later, foamy macrophages appeared and became more obvious after 2 weeks. About 2 to 5 weeks, the tissues at the necrotic site dissolved and formed cysts. The cysts which varied in size are irregular in shape and can exist in a single focus. In severe cases, multiple cysts are present. A few months later, the cyst cavity was absorbed, but the lateral ventricle enlarged or was filled with strongly proliferating astrocytes. However, not all PVL conforms to the above-mentioned development process, and the pathological changes are mainly determined by the severity of damage and brain maturity. When diffuse white matter damage occurs, it is mainly the increase of mast astrocytes and microglia, the loss of oligodendrocytes, the damage of myelination, the reduction of the overall white matter volume, and the enlargement of the ventricles, but less liquefaction occurs. Gray matter can be affected when the disease changes widely.

### 2.2. Pathogenesis

There are many causes of PVL, which are often the result of the interaction of multiple causes and multiple mechanisms. At the same time, the perinatal nervous system is in the developmental stage, and the mechanism of brain injury in premature infants is different from that in adults. Therefore, the pathogenesis of PVL is relatively complicated.

#### 2.2.1. Characteristics of Blood Vessel Development

Pathology and angiography first revealed that the main cause of white matter damage is brain tissue necrosis caused by ischemia, which is directly related to the developmental characteristics of cerebrovascular in premature infants. Long perforating branches from the anterior, middle, and posterior arteries of the brain appear at 24–28 weeks of pregnancy and extend to the edge of the ventricle to ensure the blood supply of the deep white matter around the ventricle. 32–40 weeks of gestation is the most active period for the development of a short perforator, which meets the blood supply of subcortical white matter. The anastomotic branch between the long perforator and the short perforator does not begin to form gradually until 32 weeks of pregnancy, and the incidence of PVL decreases accordingly. It can be seen that, within a period of time after the birth of premature infants, the small arteries that supply white matter have not fully developed in the anatomical structure of the premature infant.

The periventricular white matter is located at the junction and terminal area where the blood supply of the intracerebral arteries is located. When the systemic blood pressure decreases, the cerebral perfusion pressure decreases, the cerebral blood flow decreases, and the blood supply in this area decreases first and is vulnerable to ischemic damage.

#### 2.2.2. Damage to the Autoregulation of Cerebral Blood Vessels

PVL caused by cerebral blood flow regulation dysfunction can be either ischemic or hemorrhagic. The white matter of the brain is at the end of the blood supply of the internal cerebral arteries and is the lowest area of cerebral blood flow. Intracranial blood is redistributed during hypoxia-ischemia, local cerebral ischemia, shallow blood flow, and stasis and cannot recover quickly after ischemia-reperfusion preischemic state and low reactivity. During hypercapnia, the increase in cerebral blood flow is very limited. Therefore, it is easy to cause ischemic damage during hypotension and circulatory insufficiency. In addition, the vascular regulation mechanism of premature infants is not yet mature, such as the lack of smooth muscle in the perforating branch of the cerebral artery, which is prone to pressure passive cerebral circulation. Therefore, when the blood flow is abnormally increased, it is easy to cause cerebral hemorrhage. According to statistics, nearly 26% of PVL has periventricular-intraventricular hemorrhage.

#### 2.2.3. Susceptibility of Oligodendrocyte Precursors to Ischemia

Another important cause of white matter damage in preterm infants is that the developing oligodendrocyte precursors are more susceptible. Oligodendrocytes are an important component of the myelin sheath on the axons of nerve fibers.

Oxygen-free radicals are involved in the occurrence and development of brain white matter damage after asphyxiation in premature infants, mainly through damage to oligodendrocyte precursors. During brain development, the precursor cells of oligodendrocytes have obvious metabolic characteristics.

The excitotoxic effect of glutamate also has a potentially important role in the pathogenesis of PVL. The cells in the periventricular white matter of premature infants are mainly oligodendrocyte precursors and immature oligodendrocytes, which are extremely susceptible to glutamate-mediated toxicity. The toxic effects of glutamate can be achieved through glutamate receptor and nonreceptor-mediated pathways. The pathway mediated by glutamate receptors is the main mechanism of hypoxic-ischemic damage to the developing white matter. Nonreceptor-mediated pathways are related to the consumption of glutathione. Hypoxia-ischemia activates a large amount of extracellular glutamate-cysteine exchange mechanism, which causes massive consumption of intracellular cysteine and impairs glutathione synthesis. The ability of cells to scavenge oxygen-free radicals decreases, causing the death of oligodendrocyte precursors after free radical attack. The schematic diagram of the principle of evaluating the developmental state of white matter based on the combination of multiparameter changes is shown in Figure 2.

### 2.3. Clinical Diagnosis

#### 2.3.1. Clinical Manifestations

Premature infants lack specific neurological symptoms and signs when the white matter of the brain is injured and are often accompanied by a variety of serious diseases throughout the body. The clinical manifestations can be nonspecific symptoms such as poor response and hypotonia. Therefore, in premature infants, it is difficult to distinguish the symptoms from other primary diseases based on clinical alone, so early diagnosis with auxiliary examination is required.

#### 2.3.2. Imaging Examination

Head ultrasound is mainly used for brain image monitoring of premature infants. It is simple and convenient to operate, has less impact on premature infants, is relatively safe for monitoring, and is convenient for bedside operations. It can be used as the first choice for early examination of white matter lesions in critically premature infants. Head ultrasound can monitor the maturity of brain development and the progress of brain injury. Focal white matter injury (i.e., typical PVL) is easier to detect, but it is less sensitive to diffuse white matter injury. Focal white matter damage is manifested as local edema in the early stage, which usually occurs 6–12 h after acute ischemia and hypoxia. Ultrasound imaging features are mainly characterized by enhanced echo of the lesion, rough and uneven. When extensive white matter damage occurs, ultrasound can show that the strong echo radiates from around the ventricle to the subcortex. Mild edema will disappear within a few days (usually within 1 week), and ultrasound images will recover. The more severe the edema is, the more likely it will be liquefaction and necrosis and the more severe the brain damage will be. Cranial ultrasound is more sensitive to early white matter edema, but the missed diagnosis rate for white matter lesions without cyst formation is higher. In recent years, with the continuous improvement and progress of ultrasound technology, the sensitivity and specificity have also been greatly improved, but there are still certain limitations in practical applications.

The quality of the image depends on the operator's experience and technology. Many parts are difficult to show in the image, and many brain abnormalities are difficult to find. Therefore, in recent years, the internationally recommended best method for early tissue edema display is diffusion-weighted imaging. Within a few days after white matter injury, the pathological stage dominated by edema is manifested as hyperintensity in the periventricular white matter edema area.

Head CT can show low-density regional signals in the early stage of edema of brain white matter injury, usually on the upper and outer side of the anterior horn of the lateral ventricle, but because premature infants themselves are generally unmyelinated and show low density, only in the late stage, PVL with enlarged ventricles and white matter reduction is of diagnostic significance. The application of early CT only excludes intracranial hemorrhage and other congenital diseases.

In the diagnosis of white matter injury, magnetic resonance is more sensitive than cranial ultrasound. However, due to its long operation time, high cost, the need to move early infants, and the inconvenience for critically ill early infants, the brain damage detection is not as widely used as cranial ultrasound. In focal white matter injury, short T1 signals and short T2 signals around the lateral ventricle are mainly recognized. However, it is difficult to recognize MRI in the early stage of the injury, and the high signal appears in the later stage of the injury. In diffuse brain injury, magnetic resonance imaging is difficult to identify, and DWI can show abnormal high signals to the early lesions and has a good diagnostic effect on focal and diffuse white matter damage. DWI reflects the difference in tissue structure according to the motion state of water molecules in the tissue. When the damaged brain cells develop edema, the diffusion of water molecules slows down, the apparent diffusion coefficient value decreases, and DWI shows a high signal. Then the cell ruptures, the diffusion of water molecules accelerates, and the DWI signal gradually weakens. In the early stage, the magnetic resonance signal was normal, and then the corresponding change appeared. Conventional magnetic resonance is prone to omissions in the diagnosis of early white matter damage. The MRI follow-up diagram of brain injury in premature infants is shown in Figure 3.

#### 2.3.3. Laboratory Inspection

Cytokines in the molecular mechanism of white matter damage in premature infants play an important role in the occurrence of brain damage. In the pathological examination, it was found that cytokines, such as interleukin (IL), tumor necrosis factor-*α*, and neuron-specific enolase, were highly expressed in the brain injury area, and cytokines were found in animal experiments. The time is earlier than the clinical symptoms and imaging findings. Under normal circumstances, the level of IL-6 is very low, and when brain damage occurs, the release will increase significantly. Neuron-specific enolase is a marker enzyme for neurons, and it is a protein that exists in brain neurons and neuroendocrine cells. When cells undergo damage such as ischemia and hypoxia, the structure of the cell membrane is destroyed, neuron-specific enolase is released from the cytoplasm and enters the blood circulation and cerebrospinal fluid, its level rises, the release amount is positive with the degree of brain damage, and it is a sensitive and specific indicator of brain damage.

### 2.4. Treatment

There is currently no specific treatment for PVL. In recent years, in-depth research on the etiology and pathogenesis of PVL has provided potential means and methods for the prevention and treatment of PVL.

#### 2.4.1. Prevention and Treatment of Perinatal Infection

Infection is an important factor leading to PVL. Studies have shown that the use of antibiotics for prenatal infections of pregnant mothers can reduce the risk of cystic PVL in very low birth weight infants. Therefore, timely diagnosis and treatment of various infections in the perinatal period may prevent or reduce the occurrence of PVL caused by infection.

#### 2.4.2. Monitor Cerebral Blood Flow and Maintain Cerebral Perfusion

Impaired cerebrovascular autoregulation and low cerebral blood flow in preterm infants are potential factors that cause PVL in preterm infants. The application of near-infrared spectroscopy can early detect the damage of the autonomic regulation of cerebrovascular, which is of great significance for correcting hypotension, hypovolemia, and circulatory insufficiency in time to avoid the occurrence of PVL caused by cerebral ischemia.

#### 2.4.3. Correct Hypoxemia and Prevent Obvious Hypercapnia or Hypocapnia

Hypoxia directly damages brain cells. Obviously, hypercapnia or hypocapnia can cause cerebral ischemia by generating passive pressure on the cerebral circulation. Animal experiments have shown that moderate hypercapnia or hypocapnia lasting for 1 h can induce decreased brain oxidative metabolism and brain cell apoptosis, leading to PVL. Therefore, maintaining normal oxygen saturation is of great significance for the prevention and treatment of PVL.

#### 2.4.4. Use of Free Radical Scavengers

Free radical scavengers (such as vitamin E and allopurinol) can reduce the toxic effects of free radicals on oligodendrocyte precursors, and clinical use may be beneficial to the prevention and treatment of PVL.

#### 2.4.5. Others

When PVL forms, the disease is often difficult to reverse. Children with white matter damage should be systematically included in the follow-up subjects, and problems in the development of intelligence, sports, and audiovisual and sensory functions should be discovered in time, and individualized posttreatment should be given, including a series of interventions for promoting children's intellectual development at different months of age, such as physical rehabilitation and audiovisual function training, in order to obtain a certain degree of functional recovery.

## 3. Materials and Methods

### 3.1. Research Object

We selected 102 cases of term asphyxia premature infants who were hospitalized in the NICU of the First Affiliated Hospital of a university from January 2018 to February 2019 and 30 cases of healthy term infants born in the Obstetric Department of this hospital during the same period were selected as the research objects. The gestational age of the asphyxia group was 37～41 + 5 weeks, and the weight was 2.51 kg～3.90 kg. Among them, 45 cases were in the mild asphyxia group and 17 cases were in the severe asphyxia group. Thirty-six healthy full-term infants served as the control group, with a gestational age of 37 + 1 to 41 + 3 weeks and a weight of 2.54 kg to 3.83 kg. The gestational age, birth weight, gender, and delivery method of premature infants in each group were not statistically significant. All selected subjects obtained parental informed consent.

Electrolyte disorders, hypoglycemia, intrauterine infections, genetic metabolic diseases, and other congenital diseases caused by brain damage were not included in this study.

### 3.2. Research Methods

The main equipment includes Nicolet OneTM brain function monitor (Nicolet Biomedical-VIASYS-Cardinal Health, Dublin, OH), multiparameter monitor (monitoring aEEG while monitoring heart rate, blood pressure, blood oxygen saturation, etc.), conductive paste, partial scrub, and electric shaver.

Before recording, we use 70% alcohol cotton ball to disinfect the local scalp and electric shaver to shave the hair of the premature baby (shaving the forehead to the top of both sides), apply the scrub locally to reduce the resistance, and fill the disc-shaped electrode with conductive paste.

We turn on the power first, enter the basic information such as the hospitalization number of the early birth in the Nicvue management software, and then put the amplifier head box and the connecting line into the incubator and then connect the patient electrode. In the supine position, the disc-shaped electrodes are fixed with a disposable wide cloth tape. According to the international 10–20 standard electrode placement system, we place the electrodes on the forehead (Fp1; Fp2), center (C3; C4), and parietal lobe (P3; P4) on both sides of the forehead, the distance between two symmetrical electrodes is 70 mm, the reference electrode is placed at the midpoint between CZ and PZ. The electrode is not placed at the cranial suture, hematoma, or ulcer. The resistance between the disc electrode and the scalp is <18 kΩ (resistance monitoring is continued during the entire recording process). Records that do not meet the resistance requirements are not included in the final statistical data. For example, if the resistance is more than 18 kΩ, we rewash the forehead with 70% alcohol cotton balls to the top scalp on both sides and apply the scrub locally until the resistance is <18 kΩ, and then we record filter frequency 2～15 Hz. The electrode placement and impedance test are shown in Figure 4.

The EEG signal is stored in the computer hard disk in a semilogarithmic form, and the recorded graph is represented as a spectral band (aEEG) in the form of amplitude, and the raw EEG is recorded at the same time. We record within 6 hours after birth and record as long as possible, at least 4 hours each time.

### 3.3. Diagnosis of Brain Injury

According to the premature infants' HIE diagnosis basis and clinical grade formulated by the Premature Pediatrics Group of the Pediatrics Branch of the Chinese Medical Association, those who have the following 4 items at the same time can be diagnosed, and those who cannot be determined temporarily can be regarded as suspected cases. After confirming the diagnosis, it is decided whether to be selected.

1. There is a clear history of abnormal obstetrics that can lead to fetal distress and severe fetal distress (fetal heart rate <100 beats/min, lasting more than 5 minutes, and/or amniotic fluid III degree contamination). There is a history of asphyxia during the process.
2. Severe asphyxia at birth means that the Apgar score is 1 min ≤ 3 points and continues to 5 min when it is still ≤5 points and/or umbilical artery blood gas pH ≤7.100 at birth.
3. Nervous system symptoms appear shortly after birth and continue for more than 24 hours, such as changes in consciousness (excessive excitement, lethargy, and coma), changes in muscle tone (increased or weakened), abnormal original reflexes (weakened or disappeared sucking; hug reflex), serious illness, brainstem signs (changes in respiratory rhythm, changes in pupils, and slow response to light or disappearance) and increased bregma tone may occur at times.
4. We exclude convulsions caused by electrolyte disorders, intracranial hemorrhage, and birth injuries and intrauterine brain damage caused by infections, genetic metabolic diseases, and other congenital diseases.

We refer to the diagnostic criteria for multiple organ dysfunction, and it can be diagnosed if the two items are met.

1. Brain damage: hypoxic-ischemic encephalopathy, intracranial hemorrhage, or severe intracranial pressure increase needs to be confirmed by head B-ultrasonography or CT.
2. Respiratory system: respiratory failure, pulmonary hemorrhage, or pulmonary hypertension is required to be confirmed by blood gas analysis, chest X-ray, or heart color Doppler ultrasound.
3. Cardiovascular system: occurrence of heart failure, hypoxic myocardial damage, severe arrhythmia, severe electrocardiogram changes, and cardiac color Doppler ultrasound confirmed left and right heart function abnormalities, myocardial specific isoenzymes.
4. Digestive system: gastric retention, gastrointestinal bleeding, and necrotizing enterocolitis.

## 4. Experimental Results and Analysis

### 4.1. Comparison of Continuity and SWC between the Two Groups

In the HIE group, 35.09% of the early infants showed continuous amplitude integration EEG, and the proportion of SWC was 26.21%, which was significantly lower than the 98% and 96% of the control group. The differences were statistically significant (*P* < 0.05). The amplitude-integrated EEG of HIE in early birth is mainly discontinuous, and SWC is mainly immature SWC. The continuity and SWC comparison between the two groups is shown in Figure 5.

Figure 6 is aEEG background activity in contrast to continuous normal voltage in preterm infants. It is continuous, with the upper edge of the amplitude activity band >15 uV and the lower edge >5 uV. The mature SWC is expressed as normal aEEG. It can be seen from Figure 6 that the aEEG voltage fluctuates between 5 uV and 45 uV. At about 4 hours, the maximum peak is reached.

Figure 7 shows the aEEG background activity of discontinuous voltage in HIE premature infants. Its amplitude is discontinuous, the upper edge of the amplitude activity band is >10 uV, and the lower edge is <5 uV, which is indicated as a mild abnormal aEEG. It can be seen from Figure 7 that the aEEG voltage fluctuates between 0 uV and 40 uV. It reached the maximum peak at about 4 hours. However, overall, compared with Figure 6, its aEEG voltage is relatively low.

### 4.2. Comparison of the Two Groups of Highest Voltage Amplitude and Lowest Voltage Amplitude

The highest voltage amplitude of the HIE group (observation group) was 36.52 ± 1.22 uV, which was significantly higher than 23.60 ± 2.51 uV of the control group; the lowest voltage amplitude was 5.27 ± 1.38 uV, which was significantly lower than 10.66 ± 0.86 uV of the control group. The differences were statistically significant (all *P* < 0.05). The highest voltage of HIE infants rises, but the lowest voltage drops. The comparison between the two groups of highest voltage and lowest voltage is shown in Figure 8.

Figure 9 shows the continuous low-voltage aEEG background activity in HIE premature infants. The aEEG trace shows continuous low-voltage activity, the waveform is relatively flat, and there is no typical SWC; the variation range of the trace is about <7 uV, which is indicated as a severe abnormal aEEG.

Figure 10 shows the background activities of aEEG for HIE outbreak suppression in early infants. It exhibits burst suppression activity, and the variation range of aEEG trajectory is about 5 to 8 uV, which is expressed as a severely abnormal aEEG.

### 4.3. Correlation Analysis between aEEG and HIE Premature Infant Disease Degree, SBDP, and Tau Protein Expression Level

Among the 132 cases of early birth, 31 cases of mild HIE were clinically staged, 50 cases of moderate HIE, and 51 cases of severe HIE. In the results of aEEG, 36 cases of aEEG were normal, 50 cases were mildly abnormal, and 46 cases were severely abnormal. The 30 control group aEEG classification showed normal. A correlation analysis based on Spearman's method found that the monitoring results of aEEG and HIE clinical grade were positively correlated (*r* = 0.869, *P* < 0.05), as shown in Figure 11. The monitoring results of EEG are positively correlated with SBDP protein expression level (*r* = 0.678, *P* < 0.05). The combination of aEEG monitoring and protein determination can more accurately determine the degree of HIE, the prognostic value, and the efficacy of mild hypothermia.

### 4.4. Long-Term Prognosis Analysis of the Observation Group

132 cases of early-born infants underwent aEEG examination before discharge. Among the results of the examination, there were 73 cases of normal aEEG, 41 cases of mild abnormalities, and 18 cases of severe abnormalities. At the 12-month follow-up, 12 of the 132 early-born infants had a DQ value of less than 55 points, accounting for 9.31%. The monitoring results of EEG before discharge were positively correlated with the DQ value at 12 months (*r* = 0.717, *P* < 0.05). Correlation analysis between the monitoring results of aEEG at admission and the DQ value also showed a positive correlation (*r* = 0.631, *P* < 0.05). In comparison, aEEG examination before discharge is more relevant to the prognostic analysis.  Figure 12 shows the distribution of EEG results and 12-month-old DQ values before discharge.

## 5. Conclusion

The brain damage caused by perinatal asphyxia often causes the death of premature infants and subsequent neurological development disorders such as cerebral palsy, epilepsy, mental retardation, and visual and auditory impairments, which cause a serious burden on the early infants, their families, and society. Therefore, how to diagnose brain injury in premature infants has become a research hotspot at home and abroad. aEEG background activity changes are correlated with the degree of apnea. Early infants with different degrees of apnea show different types of abnormal background activities; there is a correlation between the sleep-wake cycle and the degree of apnea. The incidence of epileptic activity in the severe asphyxia group is higher than that of other groups. aEEG background activity changes, sleep-wake cycle, epileptic activity, and HIE clinical grading are closely related: mild HIE early birth aEEG background is normal or mild abnormal; moderate and severe HIE early-born infants have a lack of sleep and wake cycles or are immature; the incidence of epileptic discharges is higher in moderate and severe HIE than mild HIE. Within 6 hours after birth, aEEG can early predict the severity of brain damage in HIE premature infants caused by perinatal asphyxia. aEEG has high sensitivity, specificity, and prognostic value for the monitoring of early-born infants with severe brain injury. As a monitoring method, EEG mainly records the spontaneous discharge activity of corresponding neurons in the brain hemispheres of the tested patient and then objectively presents the brain function. Studies have shown that the amplitude-integrated EEG of early HIE infants is mainly discontinuous, while SWC is mainly immature. There is a good correlation between the expression of EEG and biomarkers. Combining multiple methods can diagnose HIE earlier and evaluate the prognosis.

## Figures and Tables

**Figure 1:** Schematic diagram of the mechanism of PVL.

**Figure 2:** Schematic diagram of the principle of evaluating the state of white matter development based on the combination of multiparameter changes.

**Figure 3:** MRI follow-up of brain injury in premature infants.

**Figure 4:** Electrode placement and brain function monitoring.

**Figure 5:** Comparison of continuity and SWC between the two groups.

**Figure 6:** aEEG background activity control of continuous normal voltage in preterm infants.

**Figure 7:** aEEG background activity of discontinuous voltage in HIE premature infants.

**Figure 8:** Comparison of the highest and lowest voltages between the two groups.

**Figure 9:** Continuous low-voltage aEEG background activities in HIE premature infants.

**Figure 10:** aEEG background activity for HIE outbreak suppression in early births.

**Figure 11:** aEEG result distribution at admission.

**Figure 12:** EEG results and 12-month-old DQ distribution before discharge.

## Data Availability

The data used to support the findings of this study are available from the corresponding author upon request.
